The article "Indirect co-culture of osteoblasts and endothelial cells in vitro based on a biomimetic 3D composite hydrogel scaffold to promote the proliferation and differentiation of osteoblasts" was published in 2024. Journal: PLoS One.

# Indirect co-culture of osteoblasts and endothelial cells in vitro based on a biomimetic 3D composite hydrogel scaffold to promote the proliferation and differentiation of osteoblasts

**DOI:** 10.1371/journal.pone.0298689

**Published:** 2024-03-25

**Authors:** Cheng Li, Guanghui Chen, Yangyang Wang, Wenwu Xu, Minghui Hu

**Affiliations:** 1 Department of Orthopedics, Jiangsu Provincial People’s Hospital, Nanjing, Jiangsu, China; 2 Department of Orthopedics, Dongguan Tungwah Hospital, Dongguan, Guangdong, China; 3 Guangdong Medical University, Zhanjiang, Guangdong, China; 4 Department of Orthopedics, DongGuan SongShan Lake Tungwah Hospital, Dongguan, Guangdong, China; National University of Singapore - Kent Ridge Campus: National University of Singapore, SINGAPORE

## Abstract

The field of orthopedics has long struggled with the challenge of repairing and regenerating bone defects, which involves a complex process of osteogenesis requiring coordinated interactions among different types of cells. The crucial role of endothelial cells and osteoblasts in bone vascularization and osteogenesis underscores the importance of their intimate interaction. However, efforts to bioengineer bone tissue have been impeded by the difficulty in establishing proper angiogenesis and osteogenesis in tissue structures. This study presents a novel approach to bone tissue engineering, involving a three-dimensional composite hydrogel scaffold composed of sodium alginate microspheres encapsulated in type I collagen. Using this scaffold, a three-dimensional indirect co-culture system was established for osteoblasts and endothelial cells to evaluate the osteogenic differentiation potential of osteoblasts. Results demonstrate that the non-contact co-culture system of endothelial cells and osteoblasts constructed by the composite hydrogel scaffold loaded with microspheres holds promise for bone tissue engineering. The innovative concept of an indirect co-culture system presents exciting prospects for conducting intercellular communication studies and offers a valuable in vitro tissue platform to investigate tissue regeneration.

## 1. Introduction

The issue of bone defects and structural loss is affecting individuals of various age groups and is a significant obstacle to maintaining a healthy lifestyle. The causes of these issues may vary, including trauma, diseases, or aging [1]. A key challenge that requires attention is the promotion and maintenance of bone formation [2, 3]. Despite being the most commonly used method in clinical practice, autologous bone transplantation has limitations such as donor availability and related complications, resulting in patients’ suffering. The utilization of allogeneic bone is limited due to its significant antigenicity and potential problems such as disease transmission and ethical issues. Therefore, there is an urgent need to identify and develop synthetic bone repair materials capable of replacing natural bone [4, 5].

Recent research has demonstrated that bone is a highly vascularized tissue, relying on tight spatial and temporal connections between blood vessels and bone cells to maintain structural integrity [6]. Thus, angiogenesis plays a crucial role in bone development and fracture healing. Through the transportation of nutrients, oxygen, and metabolic waste, blood vessels, and vascular endothelial cells facilitate the secretion of cytokines to regulate osteoblast function and promote new bone formation [7, 8]. The close interaction between endothelial cells and osteoblasts is essential for bone vascularization and osteogenesis. The exploration of the mutual regulation between these cells presents new opportunities to improve bone growth, development, repair, and reconstruction [9]. Vascularized tissue-engineered bone is currently a widely utilized technique that involves selecting the selection of scaffold materials, incorporating the incorporation of cells and cytokines, and as well as implementing implementation of various scaffold fabrication methods [10, 11]. Amler et al. [12] successfully created an in vitro model of the human mandible using 3D bioprinting, incorporating primary human mandible-derived osteoblasts and endothelial cells mimicking the vascular system. These cells not only remained viable but also effectively differentiated over 28 days. Among these methods, hydrogels are three-dimensional polymer networks that possess a high degree of swelling and porosity, enabling the diffusion of solutes and nutrients [13]. The temporary three-dimensional scaffold, which mimics the physiological function of the extracellular matrix, is critical to maintaining cellular differentiation and constructing a structural template to fill tissue damage. Collagen, as a natural polymer hydrogel, is a primary provider of structural and mechanical support in various tissues. Numerous studies have shown that collagen hydrogels promote tissue and cell growth and attachment, and enhance bone formation by facilitating osteoblast differentiation [14, 15].

During tissue growth and development, cells undergo differentiation through predetermined programs within their specific microenvironments. Tissue engineering technology has offered new possibilities to mimic the paracrine effects of cell growth, differentiation, and intercellular communication in these microenvironments. Gel microspheres have emerged as a promising vehicle for sustained delivery of encapsulated cells and bioactive molecules [16, 17]. Among the various materials used for microsphere preparation, natural polysaccharide sodium alginate has gained significant attention owing to its high porosity, permeability, minimal mass transfer limitation, and high water content, particularly in loading and targeting drug delivery [18, 19]. Alginate-based microcapsules have been extensively utilized for cell encapsulation, culture, and expansion of various cell types such as neural cells, osteoblasts, chondrocytes, and myoblasts [20, 21]. This can be attributed to the rich biocompatibility and facile cross-linking process of alginates.

In this study, we investigated the feasibility of introducing alginate gel microspheres into type I collagen hydrogel scaffolds based on the characteristics of the bone microenvironment and the advantages of alginate materials to achieve gel-sol phase transition under mild conditions. By adjusting the composition ratio of alginate and process parameters, we successfully constructed composite hydrogel scaffolds with excellent rheological and other mechanical properties. The scaffold provides a suitable microenvironment for the co-culture of osteoblasts and endothelial cells, enabling the two cell types to achieve a non-contact three-dimensional co-culture environment in vitro. Furthermore, through in vitro experiments, we confirmed that endothelial cells can promote the proliferation and differentiation of osteoblasts in the composite hydrogel scaffold. These findings lay the groundwork for a deeper understanding of the application of in vitro intercellular paracrine effects in bone tissue engineering.

## 2. Experimental procedure

### 2.1 Preparation and characterization of composite hydrogel scaffolds

#### 2.1.1 Preparation of microspheres

The calcium alginate microspheres were synthesized by utilizing the electrostatic droplet technique. Initially, 1.5% sodium alginate solution was prepared by dissolving 250 cp of sodium alginate in deionized water (dH_2_O), which was magnetically stirred for 4 hours and then refrigerated overnight at 4°C to eliminate gas. Subsequently, the syringe containing the sodium alginate solution was attached to the electrostatic droplet generator (YD-06, Dalian Institute of Chemical Physics, Chinese Academy of Sciences). Then, at a constant speed, the sodium alginate solution was pushed into the 1.1% (w/v) CaCl_2_ (Qingdao Crystal Salt Bioscience, China) solution to form calcium alginate microspheres, after adjusting the pump speed. The equipment parameters, such as voltage, frequency, syringe needle size, pump speed, and the distance between the needle and the CaCl_2_ solution’s liquid surface, were adjusted to prepare calcium alginate microspheres with different particle sizes (350 μm, 500 μm, and 1200 μm).

#### 2.1.2 Characterization of microspheres

The morphology of alginate microspheres in each group was examined under an optical microscope (CKX41SF, Japan), and the diameters of 20 individual microspheres were measured to calculate the average diameter of microspheres. Moreover, calcium alginate microspheres were pre-frozen at -80°C for 24 hours and were freeze-dried for 72 hours to obtain calcium alginate dry spheres. Scanning electron microscopy (SIEMENS, Japan) was utilized to analyze the general morphology and surface microstructure of the calcium alginate microspheres. Before observation, a vacuum gold sputtering process was conducted for 60 to 120 seconds to increase the sample’s conductivity and prevent charge accumulation. To prepare the microspheres, FITC fluorescently labeled alginate was utilized and the morphology of the calcium alginate microspheres was examined under a confocal microscope. Additionally, the sustained-release properties of VEGF-loaded microspheres were assessed through enzyme-linked immunosorbent assay (ELISA). Specifically, 250ng/ml VEGF(Peprotech, USA) was incorporated into the sodium alginate solution to prepare VEGF-loaded microspheres as previously outlined. The microspheres were then immersed in the culture medium, and the supernatant was collected from the medium on days 0, 1, 3, 7, 14, and 28, respectively. VEGF content was measured with a VEGF ELISA kit (Peprotech, USA), and optical density was monitored using a multiwell microplate reader (Thermo, USA) at a wavelength of 450 nm. VEGF concentrations were calculated based on the protocol provided by the manufacturer, and each reading was performed in triplicate.

#### 2.1.3 Composite gel scaffold formation

Using a magnetic stirrer, rat tail type I collagen(Millipore, USA) was dissolved in 0.1% glacial acetic acid, producing a 6 mg/ml type I collagen solution. After mixing the type I collagen solution with the medium, the pH was adjusted to 7.6–8.0. Calcium alginate microspheres (well-dispersed and uniform microsphere) with a diameter of 350 μm were combined with the type I collagen solution at varying volume ratios (1:3, 1:5) to form a composite hydrogel solution. The solution was then added to a specialized mold (10 mm in diameter, 5 mm in height) and allowed to collagenize for 2 hours in a 37°C incubator, forming calcium alginate microsphere-type I collagen composite gel scaffolds.

#### 2.1.4 Characterization of the composite scaffold

Scanning electron microscopy was used to observe the surface microstructures of freeze-dried calcium alginate microspheres, pure type I collagen scaffolds, and microsphere-type I collagen composite gel scaffolds.

The rheological properties of the prepared composite hydrogel scaffolds were measured by an AR2000ex rheometer (DHR, TA Instruments) to investigate the effect of different contents of calcium alginate microspheres on their rheological behavior. The relevant procedures were selected based on the operating instructions, and the storage modulus (G’) and loss modulus (G’’) of the composite gel scaffold were measured by frequency scanning. Each group of experimental samples was repeated (n≥3 times) to obtain the average value. The calcium alginate microspheres-type I collagen composite hydrogel scaffold and pure type I collagen scaffold were each divided into 3 parallel groups. Multiple measurements of each dimension of the specimen (n = 3) were carried out using a vernier caliper, and the average value was taken. Uniaxial compression testing on the composite hydrogel scaffolds was performed using a SANS universal testing machine (Shenzhen SANS Testing Machine Co., Ltd., CMT-4204, China) equipped with a force sensor with a measuring range of 1000 N (measurement accuracy of 1 mN). The loading rate was set to a strain rate of 0.01/s. The upper and lower indenters were fixed on the testing machine, lubricated with normal saline, and the composite hydrogel scaffold was placed on the lower indenter and the force was removed to zero. The upper indenter was then lowered until it just touched the upper surface of the specimen, and a preload force of 0.2N was set. The experiment started and ended when the compression reached 50% engineering strain.

### 2.2 Cell culture

Commercially available osteoblast-like MC3T3-E1 cells (China Type Culture Collection, Shanghai, China) and human umbilical vein endothelial cells (HUVECs, China Type Culture Collection, Shanghai, China) were used in this study.

The cryopreserved MC3T3-E1 osteoblasts and human umbilical vein endothelial cells (HUVECs) were thawed and cultured in DMEM/F12 medium(Thermo Fisher Scientific, USA) supplemented with 10% fetal bovine serum and 1% penicillin/streptomycin. The cells were maintained in a 37°C incubator with 5% CO_2_ and the medium was replaced every 2 days. Upon reaching a confluency of approximately 90%, the cells were detached using trypsin and subcultured. Moreover, endothelial cells in the logarithmic growth phase after resuscitation were selected for embedding in alginate microspheres and cultured separately. In addition, To realize the cell co-culture system, two kinds of cell co-culture culture systems were first established through cell acclimation experiments, and the acclimatization medium finally determined by step-by-step acclimatization method was DMEM/F12.

### 2.3 Preparation of cell-loaded hydrogel scaffolds

A composite hydrogel scaffold loaded with cells was constructed. Therefore, endothelial cells were embedded in alginate microspheres by electrostatic droplet technology. First, the endothelial cells were thoroughly mixed with sterile sodium alginate solution to form a homogeneous mixture with a cell concentration of 4×106/ml. Calcium alginate microspheres with a particle size of about 350μm were formed by dropping into calcium chloride solution by microsphere preparation apparatus. Subsequently, the osteoblast suspension (4x10^6^ cells/ml) was embedded in type I collagen solution together with endothelial cell-loaded microspheres, which were then placed in a 37°C incubator for collagenization for 2 hours, and finally a cell-loaded composite hydrogel scaffold was formed. In addition, equal amounts of osteoblasts and endothelial cells were mixed 1:1 and directly embedded in type I collagen scaffolds as a direct co-culture control group and a type I collagen scaffold loaded with the same number of osteoblasts was set up as a negative control group.

### 2.4 Cell proliferation assay

The present study employed the CCK-8 (Dojindo, Japan) assay to evaluate the proliferation of endothelial cells and osteoblasts in the co-culture scaffolds. Co-cultivation was conducted for four time points (1, 3, 5, and 7 days) followed by aspiration of the original medium and replacement with fresh medium containing 10% CCK-8 reagent. The culture was continued at 37°C in a 5% CO_2_ incubator for three hours. After incubation, a mixed medium containing 10% CCK-8 reagent was extracted (110 μl) from each sample and transferred to a fresh 96-well plate. The absorbance was measured at 450 nm to determine cell proliferation.

### 2.5 Cell viability assay

Cell viability assays were conducted utilizing a live/dead cell viability assay kit (Invitrogen, USA) by the manufacturer’s protocols. The procedure involved immersion of cell-loaded scaffolds in a medium containing 4 mM Calcein AM (green) and 2 mM homodimer-1 (red), followed by a 30-minute incubation period at room temperature. After the staining was completed, the scaffolds were rinsed thrice with sterile PBS solution and examined using a laser scanning confocal microscope (LSCM, Japan) for image acquisition.

### 2.6 VEGF quantitative analysis test

The present study employed an ELISA kit to measure the quantity of VEGF released by endothelial cells in calcium alginate microspheres-type I collagen composite scaffolds. The VEGF content was monitored on days 0, 1, 3, 7, 14, and 28. The measurement process followed the manufacturer’s protocol utilizing an amulti-well microplate reader to monitor optical density at a wavelength of 450 nm. VEGF concentrations were computed, and each reading was conducted in triplicate.

### 2.7 Fluorescent staining of cells

In this study, we utilized the cell probe DiO to label osteoblasts and DiI to label endothelial cells. The labeling method involved adding 10 μM of DiO and DiI stock solutions to 5 mL of cell culture medium, which was then added to a culture flask containing cells at 80–90% confluence. The cells were incubated in a CO_2_ cell incubator for 30–40 minutes and subsequently rinsed three times with PBS solution. They were then digested with 0.25% trypsin solution, centrifuged at 1500 rpm for 6 minutes, and cells were collected for further experimentation. To produce a composite scaffold, the cells were mixed with gel and incubated for 7 days at 37°C and 5% CO_2_. Finally, observation and image capture were performed using a fluorescence confocal microscope.

### 2.8 Detection of alkaline phosphatase activity

The alkaline phosphatase (ALP) activity of each group of cytoscaffolds (n = 5) was evaluated by utilizing an ALP kit (Wako, Japan) in line with the manufacturer’s guidelines. To accomplish this, cytoscaffold samples (n = 5) were rinsed thrice with PBS, minced, and homogenized in PBS using a glass grinder. The resulting suspension underwent two freeze-thaw cycles, further breaking down the osteoblast cell membranes. The homogenate was then centrifuged at 5000 rpm for 15 minutes, and the ALP content was assessed by following the manufacturer’s protocol for the ALP kit.

### 2.9 Alizarin red S staining and quantification

The cell scaffolds were washed with PBS, washed twice, and then 4% paraformaldehyde for cell fixation. After the cells were fixed for 30 min, they were washed twice again. After washing, 1% Alizarin Red S (Sigma, USA) was used for staining. After staining the samples were incubated in the dark for 2 hours for observation under a microscope.

### 2.10 Real-time quantitative polymerase chain reaction (real-time PCR)

To detect the expression levels of osteogenesis-related functional genes (Runx2, OCN, MMP-2), a quantitative real-time polymerase chain reaction (qRT-PCR) was performed (Table 1). Total RNA was extracted from cells on hydrogels at each time point using RNAiso Plus (TaKaRa, Japan) and converted to cDNA using the PrimeScript™ RTMix kit (TakaRa, Japan). The expression levels of the related osteogenic gene markers were analyzed using Sybr Green through qRT-PCR. The reaction conditions included 95°C for 30 seconds, 95°C for 5 seconds, 40 cycles of reaction, and 60°C for 34 seconds. GAPDH served as the internal reference gene, and the expression levels of the osteogenic function genes were calculated by normalizing the values to those of the internal reference genes, based on the 2-ΔΔCT method.

**Table 1:** The primer sequence of qRT-PCR.

Gene	Direction	Sequence (5’–3’)
Runx2	Forward	AACAGCAGCAGCAGCAGCAG
	Reward	GCACCGAGCACAGGAAGTTGC
OCN	Forward	CAGGCGCTACCTGTATCAATGGC
	Reward	GCCGATGTGGTCAGCCAACTC
MMP-2	Forward	GCCTCTCCTGACATTGACCTTGG
	Reward	CACCACGGATCTGAGCGATGC
GAPDH	Forward	GACTGATGTTGTTGACAGCCACTGC
	Reward	TAGCCACTCCTTCTGTGACTCTAAC

### 2.11 Statistical methods

The experimental data were analyzed using SPSS V20.0 software to conduct relevant statistical analyses. Each experimental condition was repeated at least three times, and the results were presented as mean ± standard deviation. For comparisons between different groups in the experiments, a one-way analysis of variance (ANOVA) was employed. Statistical significance was determined at p<0.05, with * indicating p<0.05, ** indicating p<0.01, and *** indicating p<0.001.

## 3. Results

To simulate the co-culture environment of endothelial cells and osteoblasts in vitro, we designed calcium alginate microspheres embedded in type I collagen to form a composite 3D hydrogel scaffold. The preparation process is shown in Fig 1.

**Fig 1:** Schematic diagram of indirect co-culture system of type I collagen complex hydrogel scaffolds loaded with calcium alginate microspheres.

### 3.1 Preparation and characterization of composite hydrogel scaffolds

In this study, we utilized electrostatic droplet technology to prepare calcium alginate microspheres of varying sizes (350 μm, 500 μm, and 1200 μm) and optimized the preparation conditions to obtain uniform and size-controlled microspheres (Fig 2A1–2A3). The morphology and size distribution of the microspheres were evaluated and shown to be well-dispersed, with the 350 μm microspheres demonstrating the highest uniformity (Fig 2B). Confocal microscopy was employed to observe fluorescently labeled calcium alginate microspheres, which exhibited a uniform and plump morphology (Fig 2C). Fig 2D shows the scanning electron microscope (SEM) image of the calcium alginate microspheres, revealing a uniform morphology with a loose and rough surface structure. We also conducted a release test on VEGF-loaded alginate microspheres, ensuring that the initial amount of loaded VEGF was standardized among the groups. The results revealed that smaller particle sizes resulted in more durable and stable VEGF release (Fig 2E). Subsequently, we created a 3D composite gel scaffold by mixing 350 μm sodium alginate microspheres with pure type I collagen (Fig 2F). We further characterized the structure of the composite gel scaffold by observing the surface microstructure of the alginate microspheres, pure type I collagen scaffold, and the type I collagen composite gel scaffold loaded with microspheres. The results showed that the calcium alginate microspheres underwent shrinkage, resulting in a decrease in particle size. The surface of the pure type I collagen gel scaffold exhibited densely arranged filament-shaped objects, while the microsphere-type I collagen composite gel scaffold displayed spherical protrusions wrapped in type I collagen (Fig 2G1–2G3).

**Fig 2:** A: Optical microscope images of alginate microspheres with different diameters prepared by electrostatic droplet extrusion technology (A1: 350 μm, A2: 500 μm, A3: 1200 μm), (bar = 300 μm); B: Changes in diameter of microspheres with different particle sizes; C: Morphology of fluorescently labeled calcium alginate microspheres(bar = 200 μm); D1: Microsphere morphology under scanning electron microscope(bar = 200 μm), D2: Microsphere surface structure after magnification(bar = 20 μm); E: VEGF release test comparison between microspheres of different particle sizes; F: General shape of 3D composite hydrogel scaffold; G: Morphology under scanning electron microscope(bar = 200 μm): G1 calcium alginate microspheres, G2 pure type I collagen gel scaffold, G3 microsphere-type I collagen composite gel scaffold.

### 3.2 Effects of different composition ratios on the rheological properties of calcium alginate microsphere composite gel scaffolds

This study utilized a rheometer to investigate the impact of varying calcium alginate microsphere content on the viscoelastic properties of the composite gel. Frequency scanning curves of gel scaffolds with different microsphere quantities were obtained and analyzed. Results revealed that within the 0.1-10Hz range, the storage modulus (G’) gradually increased, consistently surpassing the loss modulus (G’’) (Fig 3A1). This observation suggests that within the measured timeframe, the microsphere Type I collagen composite scaffold retains a higher energy storage capacity compared to its energy dissipation, indicating that the gel system remains in a solid phase. The overall structural integrity of the gel system remains relatively stable throughout the entire duration of the analysis. Relative comparisons of G’ and G’’ were conducted, with the G’ of the gel scaffold increasing from 222.3±6.99Pa to 515.0±13.25Pa and the G’’ increasing from 30.06±0.55Pa to 61.72±4.38Pa (Fig 3A2 and 3A3). Notably, the G’ of the composite gel scaffold experienced a more significant increase than G’’ after 1Hz, indicating greater elasticity with increasing microsphere content. According to the findings, the combination of calcium alginate microspheres and type I collagen exhibits improved storage modulus when the volume ratio is 1:3, thereby indicating favorable elastic properties of the gel scaffold.

**Fig 3:** A:Rheological properties of composite gel scaffolds with different composition ratios A1: Frequency scanning curve; A2: Storage modulus comparison; A3: Loss modulus comparison (Control is the pure type I collagen group, A is the volume ratio of 1:5 group, B is the volume ratio 1:3 group); B: The stress-strain curve of calcium alginate microspheres-type I collagen composite hydrogel scaffold and pure type I collagen scaffold; C: Light microscope images of endothelial cells cultured in calcium alginate microspheres on day 7 (C1) and day 14 (C2). In Figure C1, the endothelial cells exhibit initial adherence and proliferation within the microspheres, forming small clusters. By day 14 (C2), the endothelial cells continue to grow, and the cell clusters have increased in size while maintaining a three-dimensional morphology (bar = 100 μm); D: Image of endothelial cells stained for live and dead cells after7 (D1)and 14(D2) days of culture in microspheres. (*, **, ***, compared with the control group at the same time point, *means p<0.05, ** means p<0.01, *** means p<0.001, and n = 3).

### 3.3 Mechanical properties of the composite gel scaffold

Osteoblasts are strategically located in bone tissue to sense and respond to external mechanical loads, thereby regulating adaptive remodeling through intercellular signaling. Notably, osteoblasts exhibit a greater responsiveness to fluid stress than to mechanical stress. Subsequently, following rheological analysis of composite gel scaffolds and considering the physiological function of bone structure [22], we have identified a subset of composite gel scaffolds with superior elastic properties. Specifically, we have selected composite gel scaffolds with a microsphere-type I collagen volume ratio of 1:3 for subsequent investigation. In this study, the mechanical properties of the prepared calcium alginate microspheres-type I collagen composite hydrogel scaffold were investigated, with a pure type I collagen hydrogel scaffold serving as the control group. Stress-strain curves were analyzed (Fig 3B), revealing that the maximum pressure of the pure type I collagen scaffold reached 0.11 MPa, while the corresponding pressure of the composite hydrogel scaffold peaked at 0.32 MPa. The incorporation of calcium alginate microspheres was found to significantly enhance the mechanical properties of the composite hydrogel scaffold.

### 3.4 Expression of biological properties of cells in hydrogel scaffolds

We chose calcium alginate microspheres of 350μm particle size to encapsulate cells. Endothelial cells were cultured in the microcapsules for 7 and 14 days, respectively, as depicted in Fig 3C1 and 3C2. After 14 days, the endothelial cells within the microcapsules aggregated and formed cell clusters, which continued to grow and proliferate in a three-dimensional manner. The particle size of the cell clusters increased with time, but during the subsequent culture, the particle size remained stable. The viability of endothelial cells within the microspheres was confirmed through live/dead staining (Fig 3D1 and 3D2).

Additionally, we co-encapsulated endothelial cells and osteoblasts in alginate microspheres and embedded them in a type I collagen scaffold, as shown in Fig 4A. We observed the gross morphology of the cell-loaded composite hydrogel scaffold and the cell co-culture under the optical microscope. Furthermore, to visualize the spatial distribution of endothelial cells (red) and osteoblasts (green), they were labeled with cell probes emitting different wavelengths and seeded into the composite scaffold. The growth of cells in the three groups of hydrogel scaffolds was observed under laser confocal fluorescence microscopy, as depicted in Fig 4B–4D and 4B1–4D1. The results indicated that in the indirect co-culture group, the two cell types existed within their microenvironment in the composite scaffold.

**Fig 4:** A: The general morphology of the hydrogel scaffold loaded with cells and the co-culture of cells under the light microscope, (bar = 100 μm); B-D: Confocal microscope images illustrating the growth and distribution of hydrogel scaffold cells. Endothelial cells are marked in red, and osteoblasts are marked in green. In Figure B (negative control group), cells are sparsely distributed. In Figure C (direct co-culture control group), both cell types exist within their microenvironments. In Figure D (indirect co-culture group), the two cell types are co-cultured, exhibiting distinct spatial arrangements and interactions. Corresponding observations under the light microscope are shown in B1-D1 (bar = 100 μm); E:The release trend of VEGF in the hydrogel scaffold; F: Analysis of the proliferation ability of osteoblasts inside the hydrogel, (bar = 200 μm).

The present study extended its focus on the examination of the VEGF factors’ secretion during the endothelial cells’ cultivation in hydrogel composite scaffolds. As depicted in Fig 4E, the cumulative release of VEGF factors initiated a phase of slow release on the third day. The capability of microencapsulated cells to secrete the VEGF factor was gradually amplified as the culture time was prolonged. Subsequent to 14 days of cultivation, the level of VEGF factor secretion remained relatively stable, indicating a noticeable slow-release impact.

Moreover, we conducted a CCK8 experiment to assess the proliferation ability of cells within the hydrogel. Our results showed that osteoblasts exhibited good proliferation capacity on the surface of the hydrogel scaffolds in all three groups. Notably, the cell growth ability in the indirect co-culture group was slightly stronger than the other two groups, but there were no significant differences in the growth curves of the cells in the three groups at days 1, 3, 5, and 7 of culture (Fig 4F). Additionally, we cultured the gel scaffolds of different groups for 7 and 14 days and performed live/dead staining. Our findings indicated that there were very few dead cells in the gel scaffolds of all three groups, and as the culture time increased, osteoblasts started to proliferate within the gel (Fig 5).

**Fig 5:** Live/dead staining images of cells co-cultured on hydrogel scaffolds on day 7 and day 14, respectively. A: negative control group, B: direct co-culture control group, C: indirect co-culture group. The images reveal the dynamic morphological changes of cells over time, with green representing live cells indicating active metabolic states and intact membrane integrity, while red indicates dead cells with compromised viability and membrane integrity. The hydrogel scaffold provides a conducive environment for cell survival and proliferation. Scale bar = 200 μm.

### 3.5 Proliferation and differentiation of osteoblasts

The proliferation and differentiation potential of osteoblasts in different scaffolds were investigated in this study by co-culturing the scaffolds for 14 and 21 days, respectively, and then observed and photographed under a microscope after staining with Alizarin Red S (Fig 6). The mineralization capacity of osteoblasts was assessed by observing the calcified area of the osteoblast the extracellular matrix. ​The results indicated that the calcification area of extracellular matrix of osteoblasts increased with time, suggesting that endothelial paracrine promotes the mineralization of MC3T3-E1 cells under indirect co-culture conditions. Furthermore, a quantitative assessment of alkaline phosphatase (ALP) released by osteoblasts cultured within the hydrogel scaffold further reinforces this perspective. (Fig 7A).

**Fig 6:** Alizarin Red S staining images of cells co-cultured on the hydrogel scaffolds on the 14th and 21st days, respectively. A: negative control group, B: direct co-culture control group, C: indirect co-culture group. The images showcase the morphological changes associated with osteogenic differentiation, with prominent mineralized nodules stained in red. The hydrogel scaffold supports the osteogenic differentiation of osteoblasts, contributing to the development of a mineralized extracellular matrix. Scale bar = 200 μm.

**Fig 7:** Osteogenic differentiation of osteoblasts within scaffolds: A: ALP release amount of osteoblasts in the hydrogel scaffold; The relative mRNA expression of osteogenic function-related genes on the 7th and 14th days of osteoblast hydrogel scaffold culture (B is the expression of RUNX2; C is the expression of OCN; D is the expression of MMP-2) (*** means P < 0.001; ** means P < 0.01; * means P < 0.05,n = 3).

The expression levels of osteoblast-related genes, including Runx2, OCN, and MMP-2, were measured using qRT-PCR to evaluate osteogenic activity (Fig 7B–7D). The results showed that the mRNA expression levels of MMP-2, OCN, and RUNX2 were significantly higher in the indirect co-culture group than in the control group (P<0.05). The findings suggested that endothelial paracrine upregulated the expression of osteoblast-related genes and enhanced the proliferation, early osteogenesis, and mineralization of osteoblasts under co-culture conditions.

## 4. Discussion

Bone tissue engineering involves the use of biomaterials and cell engineering technology to repair, reconstruct, or replace human bone tissue [23–25]. However, the complex structure and biological properties of bone tissue make it challenging for traditional two-dimensional culture systems to replicate the internal environment of bone tissue. Therefore, it is imperative to develop more complex three-dimensional culture systems. This study introduces a novel approach to bone tissue engineering, utilizing a three-dimensional composite hydrogel scaffold constructed from sodium alginate microspheres wrapped in type I collagen. The present study discovered that by cultivating osteoblasts and endothelial cells within the scaffold, a three-dimensional indirect co-culture system was established, mimicking the internal three-dimensional microenvironment of bone tissue. Notably, endothelial cells successfully promoted the differentiation of osteoblasts without any exogenous factors. The novel concept of this indirect co-culture system can serve as a valuable tool for studying cell communication and provides an in vitro tissue platform for tissue regeneration.

The use of hydrogel scaffolds allows the simulation of the microenvironment in which cells exist and can aid in the formation of a structure that resembles the extracellular matrix. Alginate is a preferred material for scaffold production due to its favorable biocompatibility, biodegradability, and adhesion properties, offering a viable option for bone injury repair [26]. In this study, we utilized electrostatic droplet technology to prepare calcium alginate microspheres of varying particle sizes [27]. The preparation process is straightforward, with mild conditions and high reproducibility. The uniformity of the alginate microspheres was confirmed via scanning confocal microscopy (Fig 2C). Analysis of VEGF-loaded alginate microspheres with different particle sizes indicated that smaller microspheres facilitated more durable and stable, but also less VEGF release (Fig 2E). Zhang et al. [28] fabricated hybrid hydrogel microspheres composed of alginate and lithium silicate, possessing a particle size ranging from 350 to 450 μm. These microspheres exhibited favorable characteristics for the sustained release of VEGF. Previous studies have suggested that spherical aggregate networks with diameters between 100–400 μm are optimal for oxygen diffusion and species exchange [20]. Therefore, by optimizing the preparation conditions, we selected 350 μm calcium alginate microspheres with high uniformity for cell encapsulation in this experiment. Our research further demonstrated that endothelial cells aggregated to form cell clusters in the microspheres, where they grew and proliferated in a three-dimensional manner, reaching a plateau stage of growth on the 14th day. Thereafter, cell activity remained relatively stable at a certain level. Kang et al. [29] previously reported the limiting effect of sodium alginate on cell growth, indicating that sodium alginate microspheres can impede cell growth and metabolism to a certain extent while providing a three-dimensional culture space for cells. However, this effect also maintains the long-term activity of cells, allowing them to exert their functions over an extended period.

Collagen molecules provide ample RGD sites [30] that promote cell adhesion and proliferation, while the introduction of sodium alginate molecules allows for the regulation of the mechanical properties of hydrogels [31]. The matrix stiffness and elastic modulus of the hydrogel play significant roles in osteoblast extracellular matrix synthesis, as well as the maintenance of osteoblast phenotype and function [32]. Accurate evaluation of viscoelastic properties is crucial for biomaterial research in regenerative medicine. Therefore, we explored the impact of varying calcium alginate microsphere contents on the rheological properties of composite gel scaffolds. The results showed that the composite gel scaffold’s G’ and G" increased with increasing microsphere content. Higher storage modulus and viscoelasticity were observed as the microsphere content increased, which significantly affected the growth, proliferation, migration, nutrient diffusion, and transfer of cells within the gel. Furthermore, we compared the mechanical properties of the prepared calcium alginate-type I collagen composite hydrogel scaffold with those of pure type I collagen scaffolds. Our findings indicate that the inclusion of calcium alginate microspheres enhances the mechanical properties of the composite hydrogel scaffold.

The majority of current research on hydrogel scaffolds primarily focuses on mimicking the mechanical properties of natural bone tissue [33, 34]. However, the network structure of the resulting hydrogel scaffold is often highly compact, which is not conducive to material exchange and the transfer of bioactive factors. This can adversely affect the biological properties of cells and hinder the repair of bone tissue. To address this issue, this study leverages the advantages of alginate material and its ability to undergo a gel-sol phase transition under mild conditions, as well as the characteristics of the bone microenvironment, to propose introducing alginate gel microspheres into type I collagen hydrogel scaffolds in a solid state. This strategy establishes an indirect co-culture system of endothelial cells and osteoblasts by embedding these two different cell types in distinct regions of the scaffold. The results of cell proliferation and live/dead staining demonstrate that the cells within the scaffolds maintain good growth ability and cell survival rates.

Moreover, we conducted an investigation into the secretion of VEGF during the culture of the endothelial cell-loaded microspheres in the scaffold. Our findings unveiled that the microspheres orchestrated a regulated and gradual VEGF release profile, resulting in a significant augmentation of VEGF secretion by endothelial cells. This effect was consistently sustained throughout the study period. Prior studies have also demonstrated the potential of microsphere-based delivery systems for VEGF. For instance, Li et al. [35] developed a heparin-gelatin microsphere system that could release 50% of the loaded VEGF within 10 days, while Zhang et al. [28] reported sustained release of VEGF microspheres for over 28 days, while preserving the biological activity of VEGF. Collectively, the microencapsulated culture system offers a promising approach to enhance the VEGF secretion capability of endothelial cells and maintain this effect during prolonged culture. These findings hold great potential for the application of VEGF in various tissue engineering and orthopedic therapies, such as promoting bone repair and regeneration to alleviate conditions like osteoporosis and fractures by enhancing angiogenesis and osteocyte proliferation [36].

Our research findings indicate that the presence of endothelial cells significantly promotes the osteogenic differentiation of osteoblasts within the hydrogel scaffold. This is manifested by enhanced expression of osteogenic markers, including proteins and mRNA, as well as an elevation in alkaline phosphatase activity. In the process of bone formation, there exists a close and reciprocal interaction between VEGF and MMP-2, which holds crucial significance for extracellular matrix degradation and tissue remodeling. Past literature [37–39] underscores MMP-2 as a pivotal metalloproteinase playing a key role in the breakdown and reshaping of the extracellular matrix. Concurrently, VEGF, through the promotion of vascular neogenesis and activation of endothelial cells, may indirectly regulate the activity of MMP-2. Our research results suggest that the interaction between VEGF and MMP-2 may constitute an integral part of the cytokine network regulating bone formation. This discovery is of paramount importance for comprehending the biological significance of cytokine interactions in osteoblast function and bone matrix formation. Future studies can delve into the specific mechanistic actions of MMP-2 and its influence on critical steps in bone formation.

The composite hydrogel scaffold, composed of sodium alginate microspheres encapsulated in type I collagen, provides a platform with the potential to create a microenvironment with varying concentrations of bioactive factors. The controlled release of factors, such as vascular endothelial growth factor (VEGF) from the alginate microspheres, adds a dimension of spatial heterogeneity to the culture system. This feature mimics the natural gradients observed in the native tissue microenvironment, where cells experience diverse signaling cues depending on their location within the tissue. The concept of a gradient environment is particularly relevant in tissue engineering, as it can influence cell fate decisions and tissue morphogenesis. By incorporating this gradient-like feature into the scaffold, the study not only contributes to the understanding of intercellular communication but also opens avenues for optimizing tissue regeneration strategies. Furthermore, the rheological and mechanical properties of the composite hydrogel scaffold, as discussed in the results, play a crucial role in maintaining the structural integrity necessary for supporting cellular activities within the gradient environment. The observed increase in storage modulus (G’) and the enhanced mechanical properties of the scaffold, especially when utilizing a specific volume ratio of microspheres, highlights the potential for tailoring the scaffold to better mimic the mechanical gradients found in native tissues.

In conclusion, the integration of a gradient-like microenvironment into the three-dimensional indirect co-culture system, as demonstrated in this study, contributes not only to the advancement of cell communication studies but also holds promise for developing tissue engineering strategies that closely replicate the complexity of native tissue environments. Further investigations into refining the scaffold design and optimizing the gradient features will likely yield insights that advance the field of regenerative medicine.

## 5. Conclusions

In this research, we designed a novel composite hydrogel scaffold. Utilizes a three-dimensional composite hydrogel scaffold constructed from sodium alginate microspheres encapsulated in type I collagen. The investigation revealed that a superior storage modulus and desirable elastic characteristics were observed in the gel scaffold when the volume ratio of calcium alginate microspheres to type I collagen was 1:3. Additionally, a three-dimensional indirect co-culture system was established by cultivating osteoblasts and endothelial cells within scaffolds to analyze the paracrine effects between these cell types. The protracted release of VEGF factors from microencapsulated endothelial cells was observed to stimulate osteoblast proliferation and differentiation through paracrine signaling. The composite hydrogel-based non-contact co-culture system of endothelial cells and osteoblasts exhibits potential for bone tissue engineering applications.
